The article "Anthrax Edema Factor Toxicity Is Strongly Mediated by the N-end Rule" was published in 2013. Journal: PLoS One.

# Anthrax Edema Factor Toxicity Is Strongly Mediated by the N-end Rule

**DOI:** 10.1371/journal.pone.0074474

**Published:** 2013-08-28

**Authors:** Clinton E. Leysath, Damilola D. Phillips, Devorah Crown, Rasem J. Fattah, Mahtab Moayeri, Stephen H. Leppla

**Affiliations:** Laboratory of Parasitic Diseases, National Institute of Allergy and Infectious Diseases, National Institutes of Health, Bethesda, Maryland, United States of America; The Ohio State University, United States of America

## Abstract

Anthrax edema factor (EF) is a calmodulin-dependent adenylate cyclase that converts adenosine triphosphate (ATP) into 3’–5’-cyclic adenosine monophosphate (cAMP), contributing to the establishment of *Bacillus anthracis* infections and the resulting pathophysiology. We show that EF adenylate cyclase toxin activity is strongly mediated by the N-end rule, and thus is dependent on the identity of the N-terminal amino acid. EF variants having different N-terminal residues varied by more than 100-fold in potency in cultured cells and mice. EF variants having unfavorable, destabilizing N-terminal residues showed much greater activity in cells when the E1 ubiquitin ligase was inactivated or when proteasome inhibitors were present. Taken together, these results show that EF is uniquely affected by ubiquitination and/or proteasomal degradation.

## Introduction

The Gram-positive bacterium *Bacillus anthracis* is the causative agent of the zoonotic disease anthrax. *B. anthracis* infections are mediated by its poly-D-glutamic acid capsule [1] and the tripartite anthrax toxin [2,3], composed of protective antigen (PA), lethal factor (LF), and edema factor (EF). PA is the receptor-binding protein that delivers LF and EF into the host cell cytosol. LF is a zinc metalloprotease that cleaves mitogen-activated protein kinase kinases and Nlrp1 [4–8], a component of the inflammasome, thereby altering key signal transduction processes. EF is an adenylate cyclase that requires binding of calmodulin to catalyze the formation of cAMP from ATP [9].

The contributions of EF to bacterial dissemination and infection have been highlighted by several groups in recent years. In whole animal imaging studies, Goossens and colleagues showed that bioluminescent *B. anthracis* producing only EF and PA directly spread to the spleen, bypassing significant growth in the draining lymph nodes [10]. Likewise, we previously showed that neutralization of EF with monoclonal antibodies significantly improved the course of capsule-deficient *B. anthracis* spore infections in mice [11].

Previous work with LF showed that it is subject to degradation within host cells in a manner consistent with the N-end rule [12]. The N-end rule describes a degradation pathway that was discovered and well characterized by Ciechanover, Hershko, Rose, Varshavsky and colleagues [13,14]. Through the action of E1 and E2 ubiquitin ligases and E3 adaptors, proteins in the eukaryotic cell are interrogated as to the identity of their N-terminal amino acid. Proteins that possess N-terminal residues classified as destabilizing are preferentially post-translationally modified at lysine residues by covalent attachment of ubiquitin, a 76-amino acid protein. These ubiquitin-tagged proteins are then targeted for degradation by the proteasome (for a succinct review, see 15).

The article "Anthrax Edema Factor Toxicity Is Strongly Mediated by the N-end Rule" was published in 2013. Journal: PLoS One.

The mature amino terminal sequences of EF and LF are MNEHYTES and AGGHGDVG, respectively. The N-terminal methionine and alanine residues are both stabilizing residues according to the N-end rule. The initial cloning of EF and LF for overexpression purposes resulted in the addition to the N-terminus of a histidine [16], which is a destabilizing residue. Additionally, the expression and purification of EF in *Escherichia coli* is typically accomplished with the addition of N-terminal affinity tags [17], which could have unintended effects on protein stability once these are delivered to the target cell cytosol. Previous work showed that the N-terminal residue of LF affects its potency [12], and we sought to determine whether EF was affected in a similar manner. However, EF had been shown to be especially sensitive to proteolysis when secreted to the supernatant of non-toxigenic strains of *B. anthracis* [18]. EF purified from such strains was truncated at the N-terminus. The creation of a strain of *B. anthracis* deficient in six extracellular proteases made expression of full-length EF possible [18]. This advance allowed us to carry out a systematic study of N-end rule effects on EF activity and toxicity in mammalian cells. Our studies show that EF activity correlates with protein stability as predicted by the N-end rule, and inhibition of ubiquitination and proteasome function increases the toxicity of unstable EF N-terminal variants. 

## Materials and Methods

### Construction of EF N-terminal variants

The plasmid pSJ136EFOS [18] was used as a template for overlap extension PCR [19] to create EF N-terminal variants. EF-(M) N is the protein having the native amino acid sequence as expressed in *B. anthracis* from the virulence plasmid pXO1, specifically, the N-terminal sequence MNEHYTES. As mentioned in the Results section, overexpression and purification of this protein under the conditions described leads to the removal of the N-terminal methionine, yielding the N-terminal sequence NEHYTES. Previously reported purification of this protein has produced material containing both MNEHYTES and NEHYTES N-termini in a 50%-50% mixture [18]. The plasmid pSJ136, the parent plasmid of pSJ136EFOS, contains the EF gene with an added NdeI site on the 5’ end, giving a mature protein sequence of HMNEHYTES in a manner similar to LF with the plasmid pSJ115 [16]. The goal of the PCR process was to create plasmids encoding proteins having all 20 amino acids at the N-terminus of EF, or **X**NEHYTES, where X is each of the 20 amino acids. This was accomplished by randomizing the first codon of EF-(M) N through the use of a degenerate codon in the primer (NNS, where N = A, C, G, or T, and S = G or C). Outer primers were GACGAGCGCTTCGGTCTTAACTG (forward) and AGCAGCCAACTCAGCTTCCTTTCG (reverse) and inner primers were GCACAGGTAATTTAGAGGTGATTCAGGCA**NNS**AATGAACATTACACTGAGAGTGATATTAAAAG (forward) and TGCCTGAATCACCTCTAAATTACCTGTGC (reverse). The resulting amplicon and vector were cut with BstXI and BamHI and ligated. Ligation products were electroporated into XL1-Blue (Agilent Technologies, Inc., Santa Clara, CA) and grown overnight at 37^°^C on LB-agar plates containing 100 µg/mL carbenicillin. Plasmid was isolated from individual colonies and sequenced. Approximately 100 colonies were screened to obtain plasmids encoding all 19 non-native N-terminal residues. These 19 variants were then successively transformed through *E. coli* strain SCS110 (Agilent Technologies, Inc.) and the non-toxigenic, non-sporulating, protease-deficient *B. anthracis* strain BH460 [18].

The article "Anthrax Edema Factor Toxicity Is Strongly Mediated by the N-end Rule" was published in 2013. Journal: PLoS One.

### Protein expression and purification

BH460 strains containing each EF N-terminal variant plasmid were grown overnight at 37^°^C in 10 mL FA medium [16] with 10 µg/mL kanamycin. Bacterial supernatants were filtered using 0.22 µm PVDF 33 mm syringe filters (Millipore, Billerica, MA), then EDTA was added to a final concentration of 0.5 mM, and the supernatants were concentrated to 500 µL using an Amicon Ultra concentrator with 10,000 molecular weight cutoff membrane (Millipore). Equal volumes of each sample were loaded onto Novex 4-20% gradient Tris-Glycine gels (Life Technologies, Carlsbad, CA) and subjected to SDS-PAGE. Gels were then stained using Coomassie blue (Bio-Rad Laboratories, Hercules, CA).

Purification of EF N-terminal variant proteins at a larger scale was accomplished very similarly to the method previously described [18]. Supernatants from batches of 1-2 L were processed by a two-column purification process instead of the previously described three-column purification. Bacterial supernatants were subjected to Phenyl-Sepharose Fast Flow (low substitution, GE Healthcare Life Sciences, Piscataway, NY), separation and ammonium sulfate precipitation as previously described. The precipitated proteins were dissolved and dialyzed into 20 mM potassium phosphate, pH 7.0, 100 mM NaCl (Buffer A). These samples were loaded onto ceramic hydroxyapatite gravity columns (Bio-Rad Laboratories) and eluted in steps of 10, 20, 30, 40, and 50% Buffer B (1 M potassium phosphate, pH 7.0, 100 mM NaCl) in Buffer A. Fractions containing EF were pooled, dialyzed into 10 mM Tris, pH 8.0, 0.5 mM EDTA, concentrated if necessary, and frozen at -80°C.

The article "Anthrax Edema Factor Toxicity Is Strongly Mediated by the N-end Rule" was published in 2013. Journal: PLoS One.

### Cell culture studies

E36 and ts20 cells [20], which are derived from Chinese hamster lung, were obtained from Dr. Jonathan Yewdell (National Institute of Allergy and Infectious Diseases). Ts20 cells harbor a temperature-sensitive E1 ubiquitin ligase enzyme that is functional at 32°C (permissive temperature) and nonfunctional at 42°C (restrictive temperature). E36 is the parental hamster cell line from which ts20 was derived. E36 and ts20 cells were grown at 32°C in 5% CO_2_ using RPMI-1640 medium supplemented with 10% fetal bovine serum, 1 mM sodium pyruvate, 2 mM GlutaMAX (all from Life Technologies), 50 µg/mL gentamycin sulfate (Lonza, Walkersville, MD), and 10 mM HEPES buffer, pH 7.3 (Quality Biological, Inc., Gaithersburg, MD). RAW264.7 (American Type Culture Collection, Manassas, VA), a mouse macrophage cell line, was grown in DMEM medium (Life Technologies) with the same additives at 37°C in 5% CO_2_ atmosphere.

For toxin studies, cells were plated at 50,000 cells per well in 100 µL medium in 96-well plates (Costar # 3596, Corning, Inc., Corning, NY) the day before toxin treatment. For studies requiring temperature shifts, cells were placed at the new temperature for 1.5 h prior to toxin treatment and maintained at that temperature during intoxication. Toxin was added to wells and after 2 h cells were lysed in Cisbio lysis buffer (Cisbio US, Bedford, MA) supplemented with 50 mM EDTA and 500 µM 3-isobutyl-1-methylxanthine (IBMX, A.G. Scientific, Inc., San Diego, CA), and cAMP detection was performed with the HTRF cAMP HiRange Kit (Cisbio) according to the manufacturer’s protocol.

### Animal studies

C57BL/6J mice (n=5/group, female, 8-12 weeks) were purchased from Jackson Laboratories (Bar Harbor, ME). Mice were intravenously administered equal masses of PA and EF (e.g., 25 µg PA + 25 µg EF). Animals were monitored at 5 h, 7.5 h, 12 h and every 8 h for 7 days for malaise or death. Malaise grades of 0-3 were assigned to each mouse based on observing posture, lethargy, coat, respiratory rhythm, movement, response to stimuli and general activity in accordance to clinical disease progression scores approved by the Animal Care and Use Committee of the National Institute of Allergy and Infectious Diseases. In experiments where mice were administered bortezomib in combination with PA and EF, 20 µg bortezomib was injected intravenously 30 min prior to toxin administration by the same route and animals were monitored every 4-6 h post-challenge for malaise or death. All animal experiments were performed using protocols approved by the Animal Care and Use Committee of the National Institute of Allergy and Infectious Diseases, National Institutes of Health. 

The article "Anthrax Edema Factor Toxicity Is Strongly Mediated by the N-end Rule" was published in 2013. Journal: PLoS One.

## Results

### Characterization of EF N-terminal variants in cultured cells

Previous work had suggested that the identity and integrity of the N-terminal sequence of EF may affect its *in vivo* activity [18], similar to the situation with LF [12]. We set out to explore this hypothesis more rigorously by making EF variants having each of the 20 amino acids at the N-terminus. We accomplished this by randomizing the N-terminal codon and sequencing individual colonies until all 19 non-native variants were isolated. The 20 variant EF proteins were expressed using the plasmid pSJ136, which uses the PA promoter and signal sequence to drive expression and secretion of EF. All proteins were expressed in *B. anthracis* strain BH460, where typical yields of pure EF are 5-10 mg/L culture. Gel electrophoresis and Coomassie blue staining of concentrated supernatants showed that 18 of 20 variants expressed full length protein (Figure 1A). The variants with N-terminal proline or isoleucine did not produce full-length EF, perhaps because signal peptidases could not cleave next to these amino acids in the context of the EF protein sequence. The isoleucine N-terminal variant displayed breakdown products not seen for the other variants, for unknown reasons. All other variants had similar expression levels.

**Figure 1:** Expression and cAMP production of EF N-terminal variants. (A) SDS-PAGE of concentrated bacterial supernatants from BH460 cells secreting the 20 N-terminal EF variants. The single letter designation for each amino acid is displayed above its respective lane. (B) EF N-terminal variants in concentrated bacterial supernatants were incubated with RAW264.7 cells and 500 ng/mL purified PA with 500 µM IBMX for 2 h at 37°C before lysis and cAMP measurement. Error bars denote standard deviation. White bars denote stabilizing N-terminal amino acids, black bars denote primary destabilizing residues, dark grey bars denote secondary destabilizing residues, and light grey bars denote tertiary destabilizing residues as dictated by the N-end rule pathway. Statistical significance is denoted as summarized from Bonferroni’s multiple comparison test after a one-way ANOVA of the reciprocally transformed data. Transformation of the data was necessary due to significantly different variances of the individual data sets.

The article "Anthrax Edema Factor Toxicity Is Strongly Mediated by the N-end Rule" was published in 2013. Journal: PLoS One.

These same bacterial supernatants containing the EF N-terminal variants were then assessed for induction of cAMP in RAW264.7 cells in the presence of PA. Despite uniform levels of protein expression, there was significant variation in the levels of cAMP produced by the 18 different EF N-terminal variants (Figure 1B). Variants that contained amino acids known to be stabilizing from the N-end rule yielded the greatest amounts of cAMP production (serine, valine, alanine, glycine, and methionine), while primary destabilizing residues (lysine, arginine, histidine, phenylalanine, and tryptophan) and secondary destabilizing residues (aspartic acid and glutamic acid) produced much lower levels of cAMP. Tertiary destabilizing residues (glutamine, asparagine, and cysteine) produced intermediate levels of cAMP, as did the threonine, leucine, and tyrosine N-terminal variants. These data showed that the *in vivo* potency of EF is strongly dependent on the N-terminal residue, consistent with the N-end rule (Figure 1B).

Six of the EF constructs were selected for scale-up and purification (EF-(M) N, EF-A, EF-C, EF-H, EF-D, and EF-R). These variants were chosen to give a wide range of adenylate cyclase activities based upon the results obtained using the bacterial supernatants. Mass spectrometric analysis of the purified EF N-terminal variants (Table 1) showed that all proteins were full length, with the exception of EF-M(N), which was 125.7 mass units lighter than expected, suggesting loss of the N-terminal methionine, which was verified by N-terminal sequencing. This could possibly be explained by the removal of the N-terminal methionine by a methionine aminopeptidase after secretion into the culture medium. Removal of the N-terminal methionine resulted in an EF variant with the N-terminal sequence of NEHY, where the N-terminal asparagine is a tertiary destabilizing amino acid according to the N-end rule. This purified protein will be referred to as EF-(M) N to maintain consistency in the naming scheme of the EF N-terminal variants.

**Table 1:** Analysis of purified EF N-terminal variants by electrospray ionization mass spectrometry (ESI-MS).

Protein	Calculated Mass	MS Result	Δ
EF-(M)N	88821.7	88696	-125.7
EF-A	88761.5	88752	-9.5
EF-C	88793.6	88801	7.4
EF-H	88827.6	88822	-5.6
EF-C	88805.6	88802	-3.6
EF-R	88846.7	88850	3.3

Proteins have the N-terminal sequences XNEHYTES, where X is the residue listed, e.g., A. The exception is EF-(M) N, which has the expected sequence of MNEHYTES, and the actual sequence of NEHYTES.

The article "Anthrax Edema Factor Toxicity Is Strongly Mediated by the N-end Rule" was published in 2013. Journal: PLoS One.

Characterization of these six purified EF variants on RAW264.7 cells produced results consistent with the previous supernatant experiments (Figure 2). EF variants with histidine, aspartic acid, or arginine at the N-terminus were lower in activity than variants harboring cysteine, asparagine, or alanine as the first residue.

**Figure 2:** Production of cAMP by purified EF N-terminal variants in RAW264.7 cells. Dilutions of EF N-terminal variants were incubated with 500 ng/mL PA on RAW264.7 cells for 2 h at 37°C before lysis and cAMP measurement. The concentration of EF estimated to induce 50 nM of cAMP production is presented here.

### Inhibition of ubiquitination increases EF activity in cultured cells

As the activity of N-terminal EF variants appeared to correlate well with predicted N-end rule stability, we sought a method to directly implicate ubiquitination in the large variations observed in EF activity. The Chinese hamster lung cell mutant ts20 has a heat-sensitive E1 ubiquitin activating enzyme, so that all ubiquitin activation and transfer are prevented at 42^°^C [20]. We treated ts20 cells and their parental strain E36 with a concentration range of EF in the presence of constant PA at the permissive and restrictive temperatures. From the resulting cAMP response data, we interpolated the concentration of EF necessary to generate 50 nM cAMP in the cells under the assay conditions (Figure 3). At the permissive temperature (32^°^C), both ts20 and E36 cells displayed profiles of cAMP generation by the panel of purified EF variants very similar to that previously observed with RAW264.7 cells (compare Figure 3 and Figure 2). Likewise, the parental E36 cells showed this expected profile of cAMP levels at 42^°^C. Comparison of the most and least active EF variants under each of these conditions showed they had >100-fold difference in activity. However, upon inactivation of the E1 ubiquitin-activating enzyme in ts20 cells at 42°C, all EF variants showed high cAMP production, with only about 1 ng/mL needed to produce 50 nM cAMP. For the normally low activity EF variants, this corresponded to a >100-fold increase in potency. This confirms the view that the destabilizing EF N-terminal variants are attenuated by ubiquitination in the cytosol, and that their activity follows the N-end rule. This data also shows that similar levels of EF are translocated into the cytosol of host cells, regardless of the N-terminus.

**Figure 3:** Prevention of ubiquitination enhances cAMP production of destabilized EF variants. E36 and ts20 cells were treated with different concentrations of purified EF N-terminal variants with 500 ng/mL PA at either 32°C or 42°C for 2 h before lysis and cAMP measurement. The concentration of EF estimated to induce 50 nM of cAMP production is presented here.

The article "Anthrax Edema Factor Toxicity Is Strongly Mediated by the N-end Rule" was published in 2013. Journal: PLoS One.

### In vivo activity of EF N-terminal variants

EF N-terminal variants were tested in mice to determine whether the N-end rule effects seen in cultured cells also occur *in vivo*. EF variants injected along with PA (25 µg each component, Figure 4A) produced varying degrees of toxicity that correlated with levels of cAMP production in cultured cells. Animals administered EF variants that have primary or secondary destabilizing amino acids at the N-terminus (EF-H, EF-D, or EF-R) survived the treatment, while all animals administered an EF variant with a stabilizing N-terminal amino acid (EF-A) succumbed by 12 h (Figure 4A) and showed advanced malaise by 5 h (Figure 4B). Mice injected with EF variants containing a tertiary destabilizing amino acid (EF-(M) N, or EF-C) showed more advanced signs of malaise at later times relative to the mice challenged with EF-A (Figure 4B), and also succumbed with a delay, between 36 and 54 h (Figure 4A). Administration of a higher dose of toxin (75 µg EF + 75 µg PA, Figure 4C) resulted in death by 12 h of all mice treated with EF variants having stabilizing or tertiary destabilizing N-terminal residues (EF-A, EF-(M) N, and EF-C). Toxicity of EF-H, having a primary destabilizing residue, was delayed relative to these other three EF variants, with all animals succumbing by 76 h (Figure 4C). All animals challenged with primary or secondary destabilizing N-terminal variants (EF-R or EF-D) survived the high dose (Figure 4C) and exhibited minimal malaise symptoms (Figure 4D).

**Figure 4:** Effects of EF N-terminal variants on C57BL/6J mice. Kaplan-Meier survival curves (A, C) and malaise rating (B, D) for mice injected intravenously with 25 µg PA + 25 µg EF (A, B) or 75 µg PA + 75 µg EF (C, D). Open circles denote living mice, and black circles denote mouse death. Animals listed as dead at a given time point were removed from successive observations.

### Proteasome inhibition increases EF activity in vivo

We next tested the effect of proteasome inhibitors on EF activity *in vivo*. Mice were treated with 20 µg bortezomib 30 min prior to challenge with EF-R and EF-D (+PA) at the 75 µg dose previously shown to be nonlethal. Both toxins caused death of all mice that were pretreated with bortezomib, while not affecting the control mice (Figure 5). The times to death seen with the toxin and bortezomib combination, 500-1000 min, are comparable to those caused by EF variants possessing more stable N-terminal residues (see EF-A, Figure 4C). These results are consistent with the data above from E1 inactivation in showing that the ubiquitin-proteasome system strongly decreases potency of EF variants having destabilizing N-termini. 

The article "Anthrax Edema Factor Toxicity Is Strongly Mediated by the N-end Rule" was published in 2013. Journal: PLoS One.

**Figure 5:** Proteasome inhibition enhances toxicity of destabilized EF variants in vivo. C57BL/6J mice were injected intravenously with 20 µg bortezomib 30 min prior to challenge with 75 µg of EF N-terminal variants+75 µg PA. Animals were monitored every 4-6 h for signs of malaise and/or death. Open circles denote living mice, and black circles denote mouse death.

## Discussion

In this work, we show that EF activity correlates well with predicted N-end rule stabilities. We also show that loss of ubiquitination in cells with a temperature-sensitive E1 enzyme greatly increases the activity of unstable EF variants, and likewise, inhibition of proteasome function with bortezomib *in vivo* increases the toxicity of unstable EF variants.

Proteins in the cell undergo the process of ubiquitination by the covalent linkage of ubiquitin to a lysine of the protein of interest. This transfer is accomplished by the formation of an amide bond between the amino group of a lysine side chain and the carboxy terminus of ubiquitin [13]. EF is potentially an excellent target for ubiquitination because it possesses 101 lysines in the mature protein, and each one is solvent accessible [21]. This is 13.2% of the 767 total residues in EF. Eleven of these lysines interface directly with calmodulin when the two proteins form a complex, including two lysines that are involved in hydrogen bonds and another two that form salt bridges. There is also a lysine in the active site, and its mutation to arginine has been shown to abrogate EF activity [22].

Previous work with LF showed that there is an approximately six-fold difference in toxicity observed in RAW264.7 cells between LF N-terminal variants [12]. This stands in contrast to the results obtained here with EF, where there was a >100-fold difference between the efficacies of the destabilized and most stable variants. The prevalence of lysine in LF (10.7% of all residues) is not vastly different from that of EF, but EF requires the binding of the cytoplasmic protein calmodulin to reconstitute its activity while LF has no such requirement. It is quite likely that ubiquitination of EF can prevent calmodulin binding and subsequent activation, resulting in the dramatic differences in activity of these EF N-terminal variants. Thus, inactivation would follow mono-ubiquitination and would not depend on poly-ubiquitination or proteasomal degradation.

We have shown that the inhibition of ubiquitination in cells expressing a temperature-sensitive E1 ubiquitin ligase and inhibition of proteasome degradation by bortezomib result in increased cAMP levels and toxicity, presumably by stabilizing EF. In contrast, proteasome inhibition had a protective effect on rats treated with LF [23], an effect paralleled by the ability of proteasome inhibitors to protect mouse macrophages exposed to LF [24]. While it is likely that inhibition of the proteasome is actually stabilizing LF against degradation, this effect is masked in the rat model of intoxication, where the Nlrp1 inflammasome, the activation of which requires proteasome activity [25], controls animal sensitivity to that toxin [8].

The article "Anthrax Edema Factor Toxicity Is Strongly Mediated by the N-end Rule" was published in 2013. Journal: PLoS One.

Previous work has shown that EF appears to be quite sensitive to degradation when overexpressed in *B. anthracis*. Expression of full-length EF was accomplished only through the construction of a strain deficient in six proteases [18]. In these studies, the expression of each protein was relatively equal across all samples, with the exception of variants with isoleucine and proline at the N-terminal position of the mature protein. While the effect of isoleucine on the lack of expression is unclear, it is known that a proline at the cleavage site will inhibit signal peptidase in *E. coli* [26,27]. It is likely that a similar response would be observed in Gram positive organisms such as *B. anthracis*.

Mass spectrometric data indicated that a methionine aminopeptidase is acting on the wild type EF-(M) N (N-terminal methionine) variant when overexpressed in culture and purified as described. All other EF N-terminal variants that were purified yielded mass spectrometric analyses that were consistent with their expected molecular weights. Moreover, the N-terminal methionine variant was confirmed by Edman degradation sequencing to lack its N-terminal methionine. The removal of this N-terminal methionine is consistent with previously published purifications of EF-(M) N from *B. anthracis* strain BH460, where a mixture of full-length and the methionine-deficient EF was observed [18]. There are four annotated methionine aminopeptidases in *B. anthracis*, inferred from homology to *B. subtilis* methionine aminopeptidases. These are all expected to be cytoplasmic proteins, but it is possible that lysis of some cells liberated enough methionine aminopeptidase to process all of the EF. Otherwise, there might be a heretofore unidentified methionine aminopeptidase that is secreted, and this is acting on EF.

The results presented here also have biotechnological applications that go beyond the understanding of effects of ubiquitination and degradation on EF toxicity. First, EF in combination with PA can be used to intoxicate a multitude of cells, making these EF N-terminal variants excellent tools for high throughput screening of the ubiquitin and proteasome degradation pathways. With differences exceeding 100-fold between the most stable and destabilized EF variants at a 2-h time point, this assay is extremely sensitive and rapid. In conjunction with EF, the cAMP detection assay is highly useful because it is quick, robust, and fully optimized for 96-, 384-, and 1536-well assays. Additionally, the ability to produce consistent batches of EF that are as potent as the native protein released during anthrax infection will facilitate studies on *in vivo* EF function and lead to a greater understanding of its effects in the host. It is also advantageous because over-production of highly active EF from its native species eliminates possible lipopolysaccharide (LPS) contamination due to expression and purification from *E. coli*. This has become increasingly important as the effects of EF in anthrax disease are being recognized as more important than previously appreciated, perhaps rising in importance to the level of LF.

The article "Anthrax Edema Factor Toxicity Is Strongly Mediated by the N-end Rule" was published in 2013. Journal: PLoS One.

## References

[1] FouetA (2009) The surface of *Bacillus anthracis* . Mol Aspects Med 30: 374-385. doi:10.1016/j.mam.2009.07.001. PubMed: 19607856.1960785610.1016/j.mam.2009.07.001

[2] MoayeriM, LepplaSH (2009) Cellular and systemic effects of anthrax lethal toxin and edema toxin. Mol Aspects Med 30: 439-455. doi:10.1016/j.mam.2009.07.003. PubMed: 19638283.1963828310.1016/j.mam.2009.07.003PMC2784088

[3] YoungJA, CollierRJ (2007) Anthrax toxin: receptor binding, internalization, pore formation, and translocation. Annu Rev Biochem 76: 243-265. doi:10.1146/annurev.biochem.75.103004.142728. PubMed: 17335404.1733540410.1146/annurev.biochem.75.103004.142728

[4] LevinsohnJL, NewmanZL, HellmichKA, FattahR, GetzMA et al. (2012) Anthrax lethal factor cleavage of Nlrp1 is required for activation of the inflammasome. PLOS Pathog 8: e1002638 PubMed: 22479187.2247918710.1371/journal.ppat.1002638PMC3315489

[5] HellmichKA, LevinsohnJL, FattahR, NewmanZL, MaierN et al. (2012) Anthrax lethal factor cleaves mouse nlrp1b in both toxin-sensitive and toxin-resistant macrophages. PLOS ONE 7: e49741. doi:10.1371/journal.pone.0049741. PubMed: 23152930.2315293010.1371/journal.pone.0049741PMC3495862

[6] DuesberyNS, WebbCP, LepplaSH, GordonVM, KlimpelKR et al. (1998) Proteolytic inactivation of MAP-kinase-kinase by anthrax lethal factor. Science 280: 734-737. doi:10.1126/science.280.5364.734. PubMed: 9563949.956394910.1126/science.280.5364.734

[7] KlimpelKR, AroraN, LepplaSH (1994) Anthrax toxin lethal factor contains a zinc metalloprotease consensus sequence which is required for lethal toxin activity. Mol Microbiol 13: 1093-1100. doi:10.1111/j.1365-2958.1994.tb00500.x. PubMed: 7854123.785412310.1111/j.1365-2958.1994.tb00500.x

The article "Anthrax Edema Factor Toxicity Is Strongly Mediated by the N-end Rule" was published in 2013. Journal: PLoS One.

[8] NewmanZL, PrintzMP, LiuS, CrownD, BreenL et al. (2010) Susceptibility to anthrax lethal toxin-induced rat death is controlled by a single chromosome 10 locus that includes rNlrp1. PLOS Pathog 6: e1000906 PubMed: 20502689.2050268910.1371/journal.ppat.1000906PMC2873920

[9] LepplaSH (1982) Anthrax toxin edema factor: a bacterial adenylate cyclase that increases cyclic AMP concentrations of eukaryotic cells. Proc Natl Acad Sci U S A 79: 3162-3166. doi:10.1073/pnas.79.10.3162. PubMed: 6285339.628533910.1073/pnas.79.10.3162PMC346374

[10] DumetzF, JouvionG, KhunH, GlomskiIJ, CorreJP et al. (2011) Noninvasive imaging technologies reveal edema toxin as a key virulence factor in anthrax. Am J Pathol 178: 2523-2535. doi:10.1016/j.ajpath.2011.02.027. PubMed: 21641378.2164137810.1016/j.ajpath.2011.02.027PMC3124019

[11] LeysathCE, ChenKH, MoayeriM, CrownD, FattahR et al. (2011) Mouse monoclonal antibodies to anthrax edema factor protect against infection. Infect Immun 79: 4609-4616. doi:10.1128/IAI.05314-11. PubMed: 21911463.2191146310.1128/IAI.05314-11PMC3257937

[12] GuptaPK, MoayeriM, CrownD, FattahRJ, LepplaSH (2008) Role of N-terminal amino acids in the potency of anthrax lethal factor. PLOS ONE 3: e3130. doi:10.1371/journal.pone.0003130. PubMed: 18769623.1876962310.1371/journal.pone.0003130PMC2518864

[13] HershkoA, CiechanoverA (1998) The ubiquitin system. Annu Rev Biochem 67: 425-479. doi:10.1146/annurev.biochem.67.1.425. PubMed: 9759494.975949410.1146/annurev.biochem.67.1.425

[14] VarshavskyA (1997) The N-end rule pathway of protein degradation. Genes Cells 2: 13-28. doi:10.1046/j.1365-2443.1997.1020301.x. PubMed: 9112437.911243710.1046/j.1365-2443.1997.1020301.x

[15] VarshavskyA (2008) The N-end rule at atomic resolution. Nat Struct Mol Biol 15: 1238-1240. doi:10.1038/nsmb1208-1238. PubMed: 19050717.1905071710.1038/nsmb1208-1238

[16] ParkS, LepplaSH (2000) Optimized production and purification of *Bacillus anthracis* lethal factor. Protein Expr Purif 18: 293-302. doi:10.1006/prep.2000.1208. PubMed: 10733882.1073388210.1006/prep.2000.1208

[17] FirovedAM, MillerGF, MoayeriM, KakkarR, ShenY et al. (2005) *Bacillus anthracis* edema toxin causes extensive tissue lesions and rapid lethality in mice. Am J Pathol 167: 1309-1320. doi:10.1016/S0002-9440(10)61218-7. PubMed: 16251415.1625141510.1016/S0002-9440(10)61218-7PMC1603774

[18] PomerantsevAP, PomerantsevaOM, MoayeriM, FattahR, TallantC et al. (2011) A *Bacillus anthracis* strain deleted for six proteases serves as an effective host for production of recombinant proteins. Protein Expr Purif 80: 80-90. doi:10.1016/j.pep.2011.05.016. PubMed: 21827967.2182796710.1016/j.pep.2011.05.016PMC3183367

The article "Anthrax Edema Factor Toxicity Is Strongly Mediated by the N-end Rule" was published in 2013. Journal: PLoS One.

[19] HoSN, HuntHD, HortonRM, PullenJK, PeaseLR (1989) Site-directed mutagenesis by overlap extension using the polymerase chain reaction. Gene 77: 51-59. doi:10.1016/0378-1119(89)90358-2. PubMed: 2744487.274448710.1016/0378-1119(89)90358-2

[20] KulkaRG, RaboyB, SchusterR, ParagHA, DiamondG et al. (1988) A Chinese hamster cell cycle mutant arrested at G2 phase has a temperature-sensitive ubiquitin-activating enzyme, E1. J Biol Chem 263: 15726-15731.3049611

[21] ShenY, ZhukovskayaNL, GuoQ, FloriánJ, TangWJ (2005) Calcium-independent calmodulin binding and two-metal-ion catalytic mechanism of anthrax edema factor. EMBO J 24: 929-941. doi:10.1038/sj.emboj.7600574. PubMed: 15719022.1571902210.1038/sj.emboj.7600574PMC554124

[22] XiaZG, StormDR (1990) A-type ATP binding consensus sequences are critical for the catalytic activity of the calmodulin-sensitive adenylyl cyclase from *Bacillus anthracis* . J Biol Chem 265: 6517-6520. PubMed: 2108958.2108958

[23] NewmanZL, CrownD, LepplaSH, MoayeriM (2010) Anthrax lethal toxin activates the inflammasome in sensitive rat macrophages. Biochem Biophys Res Commun 398: 785-789. doi:10.1016/j.bbrc.2010.07.039. PubMed: 20638366.2063836610.1016/j.bbrc.2010.07.039PMC2925535

[24] TangG, LepplaSH (1999) Proteasome activity is required for anthrax lethal toxin to kill macrophages. Infect Immun 67: 3055-3060. PubMed: 10338520.1033852010.1128/iai.67.6.3055-3060.1999PMC96621

[25] WickliffeKE, LepplaSH, MoayeriM (2008) Killing of macrophages by anthrax lethal toxin: involvement of the N-end rule pathway. Cell Microbiol 10: 1352-1362. doi:10.1111/j.1462-5822.2008.01131.x. PubMed: 18266992.1826699210.1111/j.1462-5822.2008.01131.xPMC2500182

[26] NilssonI, von HeijneG (1992) A signal peptide with a proline next to the cleavage site inhibits leader peptidase when present in a sec-independent protein. FEBS Lett 299: 243-246. doi:10.1016/0014-5793(92)80124-Y. PubMed: 1544500.154450010.1016/0014-5793(92)80124-y

[27] Barkocy-GallagherGA, BassfordPJJr. (1992) Synthesis of precursor maltose-binding protein with proline in the +1 position of the cleavage site interferes with the activity of Escherichia coli signal peptidase I in vivo. J Biol Chem 267: 1231-1238. PubMed: 1730647.1730647

